# Artificial Intelligence-Enabled Medical Analysis for Intracranial Cerebral Hemorrhage Detection and Classification

This article has been retracted.

**DOI:** 10.1155/2022/2017223

**Published:** 2022-03-21

**Authors:** Fanhua Meng, Jianhui Wang, Hongtao Zhang, Wei Li

**Affiliations:** ^1^Stroke Unit, The Affiliated Hospital of Beihua University, Jilin 132011, Jilin, China; ^2^Neuromedical Center, South China Hospital Affiliated to Shenzhen University, Shenzhen 518111, Guangdong, China; ^3^Medical Imaging Center, The Affiliated Hospital of Beihua University, Jilin 132011, Jilin, China

## Abstract

Intracranial hemorrhage (ICH) becomes a crucial healthcare emergency, which requires earlier detection and accurate assessment. Owing to the increased death rate (around 40%), the earlier recognition and classification of disease using computed tomography (CT) images are necessary to ensure a favourable prediction and restrain the existence of neurologic deficits. Since the manual diagnosis approach is time-consuming, automated ICH detection and classification models using artificial intelligence (AI) models are required. With this motivation, this study introduces an AI-enabled medical analysis tool for ICH detection and classification (AIMA-ICHDC) using CT images. The proposed AIMA-ICHDC technique aims at identifying the presence of ICH and identifying the different grades. In addition, the AIMA-ICHDC technique involves the design of glowworm swarm optimization with fuzzy entropy clustering (GSO-FEC) technique for the segmentation process. Besides, the VGG-19 model was executed for generating a collection of feature vectors and the optimal mixed-kernel-based extreme learning machine (OMKELM) model is utilized as a classifier. To optimally select the weight parameter of the MKELM technique, the coyote optimization algorithm (COA) was utilized. A wide range of simulation analyses are carried out under varying aspects. As part of the AIMA-ICHDC method, ICH can be detected and graded using a single sample. For segmentation, the AIMA-ICHDC technique uses the GSO-FEC method, which is the design of glowworm swarm optimization (GSO). The comparative outcomes highlighted the betterment of the AIMA-ICHDC technique compared to the recent state-of-the-art ICH classification approaches in terms of several measures.

## 1. Introduction

This research topic is a serious case with a higher rate of morbidity and mortality [1]. Without intensive and rapid medication, it might cause an increase in intracranial pressure, resulting in brain herniation or permanent brain tissue damage [2]. Intracerebral brain hemorrhage (ICH) is brain bleeding caused by a ruptured blood artery in the head. As blood volume grows, pressure build-up can result in brain injury, unconsciousness, or even death. It occurs when a blood vessel in the skull rupture. It can be caused by a catastrophic brain injury or nontraumatic causes such an aneurysm rupture. These factors increase the chance of an intracranial hemorrhage. A CT (computed tomography) scan is the only method that can be used to accurately diagnose an intracranial hemorrhage and is therefore the gold standard for diagnosis. It is necessary to cite. 3T-MRI scanning can also be used in problematic instances. More specifically, extra-axial hemorrhage consists of three subclasses: subarachnoid hemorrhage resulting from ruptures or trauma of arteriovenous or aneurysms malformation, epidural hemorrhage resulting from trauma, and subdural hemorrhage caused by tearing of the connecting veins in the subdural space. Intra-axial hemorrhage consists of two subclasses: intraventricular (inside brain's ventricles) and intraparenchymal (inside the brain tissue). Effective medical interference needs an accurate and urgent diagnosis for these serious conditions [3].

Computed tomography (CT) imaging of the brain is generally conducted in the emergency department, in the early diagnosis test for severe ICH. In CT images, the pattern of bleeding and the anatomic location indicate the possible causes of the ICH. Precise interpretation is essential as misdiagnoses (missed or ICH incorrect classification) might contain medical consequences [4]. Additionally, investigating CT images for specific locations and types of ICH by radiotherapists could be time-consuming and complicated. Delays in diagnoses have a direct impact from onset to treatment for patients with ICH that might affect health consequences [5]. An automated diagnosis method to help accurate and just-in-time diagnosis of ICH as well as classification of its subtypes is crucial to quicken the process of decision-making in medical intervention to enhance consequences. The earlier diagnosis of ICH is essential for adequate scheduling of scanning and better treatment. Hence, several studies are designing computer-assisted CAD for ICH segmentation.

The CAD system for the segmentation of ICH is depending on (i) manual segmentation where there is a requirement of experts for providing accurate input for segmentation or (ii) automated segmentation where hemorrhage is diagnosed without any medical intervention [6]. It is noteworthy that several research studies were carried out in manual segmentation and some studies were performed automated segmentation for ICH. Advancements in computer vision methods, like deep learning (DL), have proved enormous possibilities to extract significant data from healthcare images. Current developments are shown in technique as a great accomplishment in various segmentation with classification processes [7]. The CNN model, specially trained for segmentation or detection processes using prelabelled, large datasets, has progressed into promising methods for fully automated image assessments [8]. Recently, there has been some publication on the neural network that is capable of detecting and partially even classifying subtypes of ICH [9], along with estimating further pathologies, namely, midline shifts and skull fractures.

This study introduces an AI-enabled medical analysis tool for ICH detection and classification (AIMA-ICHDC) using CT images. The proposed AIMA-ICHDC technique initially eradicates the noise using the median filtering (MF) technique. After that, image segmentation using glowworm swarm optimization with fuzzy entropy clustering (GSO-FEC) technique is applied. Moreover, VGG-19-based feature extraction with an optimal mixed-kernel-based extreme learning machine (OMKELM)-based classifier was used. Furthermore, the coyote optimization algorithm (COA) is employed for the parameter tuning process. In order to report the betterment of the AIMA-ICHDC technique, a comprehensive set of simulations are implemented using the benchmark ICH dataset.

## 2. Related Works

Joo et al. [10] proposed a DL method for automatic localization and detection of accuracy. Afterward automatic ground truth segmentation of aneurysm, a DL method-related three-dimensional ResNet frameworks are determined by the trained set. Its specificity, sensitivity, and positive predictive values are estimated in the external and internal test set. Kim et al. [11] proposed a CAD scheme for smaller-sized aneurysm ruptures with the help of CNN-based image of 3D digital subtraction angiography. A retrospective dataset that includes 368 persons has been utilized as trained cohorts for CNN with the TensorFlow framework. An aneurysm image in six directions is attained in all the patients, and the ROI in all the images has been extracted.

Jnawali et al. [12] developed a fully automatic DL architecture that learns to identify brain hemorrhage-based cross-sectional CT images. First, the presented method extracts features by utilizing three-dimensional CNN and detecting brain hemorrhage with the help of logistic function as the final layers of the network. Lastly, developed an ensemble of three distinct three-dimensional CNN frameworks for improving the classification performances. Shi et al. [13] presented a DL-based method has better understanding of the quality of image and is verified with distinct manufacturers. The experiments are carried out in external and internal cohorts consecutively, where it attains an enhanced lesion- and patient-level sensitivity. Chen et al. [14] proposed an AI algorithm to enhance the performance of magnetic induction tomography (MIT) inverse problem. The DL systems, involving DAE, RBM, DBN, and SAE, are utilized for solving the nonlinear recreation problems of MIT and compared the recreation outcomes of DL networks.

Solorio-Ramírez et al. [15] proposed a pattern classification technique, based on Minimalist Machine Learning (MML) implementation and a highly relevant feature selection method, so-called dMeans. Phan et al. [16] developed a method-based DL and Hounsfield unit systems. It describes the duration and level of hemorrhage as well as classifies the brain hemorrhagic region on the MRI image. From the experiment, we evaluated and compared three NN systems for selecting the relevant method for classification.

## 3. The Proposed Model

In this study, an effective AIMA-ICHDC technique has been developed for the classification and recognition of ICH using CT images. The AIMA-ICHDC technique encompasses several subprocesses such as preprocessing, segmentation, feature extraction, MKELM-based classification, and COA-based parameter optimization. The design of the GSO algorithm for improving the efficiency of the FEC technique and COA to tune the parameters of the MKELM technique helps for accomplishing enhanced ICH classification performance.  Figure 1 illustrates the process of the proposed AIMA-ICHDC technique.

### 3.1. MF-Based Preprocessing

Firstly, the CT images are preprocessed using MF technique to get rid of the noise that exists in them. MF according to their specificity is one of the applications from clinical image noise extraction [17]. An important idea behind MF is for presenting *m* × *n* neighborhood for assembling every neighborhood from the increasing order. This approach was demonstrated by the subsequent formula:

(1) $$\begin{array}{c} y_{\left(m,n\right)}=\text{median}\left\{x_{\left(i,j\right)},\left(i,j\right)\in C\right\},\; \end{array}$$

where *C* indicates the centered neighborhood nearby place (*m*, *n*) of an image. During this case, an MF was implemented to digital noise extraction from the CT image.

### 3.2. Image Segmentation Using GSO-FEC Technique

During the image segmentation process, the GSO-FEC technique has been derived to identify the abnormal regions in the image. The FEC technique presented by Tran and Wagner [18] is a different generalized hard *c*‐means (HCM) clustering technique that gets benefits of fuzzy entropy. Assuming that *X* = (*x*_1_, *x*_2_,…, *x*_*N*_) are pictures with *N* pixels, and that *x*_*j*_ denotes the feature of the*j*thpixel, this technique allows for the separation of an image with the main purpose minimised in terms of a distinct matrix *U* = (*u*_*ij*_)_*C*×*N*_ and a*C* cluster prototype *C* = (*c*_*i*_)_*C*_ with 1 < *C* < *N*.The typical FEC main purpose is provided as

(2) $$\begin{array}{c} J_{\text{FEC}}\left(X,C,U\right)=\sum_{i=1}^{C}\sum_{j=1}^{N}u_{ij}d^{2}\left(x_{j},\;c_{i}\right)+n\sum_{i=1}^{C}\sum_{j=1}^{N}u_{ij}\text{log }\left(u_{ij}\right).\; \end{array}$$

It must fulfil the subsequent states:

(3) $$\begin{array}{c} U\in \left\{u_{ij}\in \left[0,1\right]|\sum_{i=1}^{C}u_{ij}=1,\;\forall j\text{ and }0\sum_{j=1}^{N}u_{ij},\;\forall i\right\}, \end{array}$$

where *x*_*j*_ refers the feature of the *j*th pixel from the image, that is, the intensity value or gray values; *d*^2^(*x*_*j*_, *c*_*i*_) represents the feature *x*_*j*_ and the cluster center *c*_*i*_. The Picard iteration was executed for solving this issue. The FEC main purpose, *J*_FEC_, is iteratively minimizing by utilizing the subsequent upgrade formulas:

(4) $$\begin{array}{c} u_{ij}={\left\{\sum_{r=1}^{C}{\left[e^{d^{2}\left(x_{j},c_{i}\right)-d^{2}\left(x_{j},c_{r}\right)}\right]}^{1/n}\right\}}^{-1},\\ c_{i}=\frac{\left[\sum_{j=1}^{N}u_{ij}x_{j}\right]}{\left[\sum_{j=1}^{N}u_{ij}\right]}. \end{array}$$

Once the technique is converged, a defuzzification procedure occurs for converting the partitioning matrix *U* to crisp separation. Generally, the maximal membership process technique that allocates the pixel *j* to cluster *C*_*i*_ with maximum membership was implemented as

(5) $$\begin{array}{c} C_{i}=\text{arg}\left\{\text{max}\left\{u_{ij}\right\}\right\},\;\text{with }i=1,2,\ldots ,C. \end{array}$$

Asuming the primary goal,*J*_FEC_(2), once it can be assumed cluster as fuzzy set. Therefore, minimized *J*_FEC_ denotes the concurrently minimized dispersion from the cluster and maximized amount of membership of the member. But, this main function does not obtain as to account for some spatial data with bias alteration. This metric considers that all features of data points were similarly vital and independent of each other, and based on clusters with spherical shapes. This statement could not be continuously fulfilled in real applications, particularly from the image clustering segmentation.

In order to avoid the local optima problem of the FEC technique, the GSO algorithm has been utilized. GSO is an advanced swarm intelligence approach presented by Pham and Kavitha [19, 20]. GSO was initially utilized to optimize multimodal functions with uneven or equivalent plan function values. In GSO, *S* glowworm swarm comprises *m* glowworm, which is dispersed in the objective function search space. All the glowworms *g*_*j*_(*j* = 1,…, *m*) is allocated an arbitrary location *p*_*j*_ within the provided function search space. Glowworm *g*_*j*_ carries its own luciferin level *L*_*j*_ as well as has the vision range named as local decision range *rd*_*j*_. The luciferin level is based on the glowworm position and main function values. The glowworm with an optimum location is brighter than others, and then, it has high luciferin level values and is closer to the best possible solution. Each glowworm seeks the neighborhood set with the limited decision range and moves to the brighter one inside the neighborhood set. In the beginning, each glowworm carries an equivalent luciferin level (*L*_0_). The *r*  *d* and radial sensor range *r*_*s*_ are initiated with the same values (*r*_0_). Next, the iteration method comprises various luciferin upgrades and glowworm movement is implemented to detect the best possible solution. All over the luciferin level updates, the objective function is estimated at the present glowworm location (*p*_*j*_) and the luciferin levels for each glowworm are utilized for the new objective function value. The *L*_*j*_ luciferin levels are upgraded by

(6) $$\begin{array}{c} L_{j}\left(t\right)=\left(1-\rho \right)L_{j}\left(t-1\right)+\gamma F\left(p_{j}\left(t\right)\right), \end{array}$$

where *L*_*j*_(*t* − 1) represent the preceding luciferin level for glowworm *j*; *γ* indicates the luciferin enhancement fraction; *p* indicates the luciferin constant (*ρ* ∈ (0,1)), and *F*(*p*_*j*_(*t*)) signifies the glowworm *j* at present location (*p*_*j*_); and *t* denotes the present iterations. Next, all the *j* glowworms explore their own neighborhood regions for extracting the neighbor that has the maximum luciferin levels by using the subsequent rules [21]:

(7) $$\begin{array}{c} z\in N_{j}\left(t\right)\text{,}\;\text{iff }d_{jz}<rd_{j}\left(t\right)\text{ and }L_{Z}\left(t\right)>L_{j}\left(t\right), \end{array}$$

where *d* indicates the distance and *Z* represents the nearer glowworm to glowworm *j*, *N*_*j*_(*t*) implies the neighborhood set, *d*_*jz*_ indicates the Euclidean distance among glowworms *j* and *z*, *rd*_*j*_(*t*) signifies the local decision range for *j* glowworm, and *L*_*Z*_(*t*) & *L*_*j*_(*t*) indicate the luciferin level for glowworm *z* and *j*, respectively. Next, to choose the optimal neighbors from the neighborhood setting, the probability for each neighbor is estimated by

(8) $$\begin{array}{c} {\text{prob}}_{jz}=\frac{L_{Z}\left(t\right)-L_{j}\left(t\right)}{\sum_{k\in N_{j}\left(t\right)}L_{k}\left(t\right)-L_{j}\left(t\right)}. \end{array}$$

Let *z* be the neighborhood set *N*_*j*_(*t*) of glowworm *j*. Later, all the glowworms select the direction of motion by the roulette wheel methodology where the glowworm with the high chance has a high possibility to be elected from the neighborhood set.  Figure 2 depicts the flowchart of GSO technique.

Later, the glowworm location (*p*_*j*_) is altered according to the elected neighbor location (*p*_*z*_) as follows:

(9) $$\begin{array}{c} p_{j}\left(t\right)=p_{j}\left(t-1\right)+s\frac{p_{z}\left(t\right)-p_{j}\left(t\right)}{{\text{Distance}}_{jz}}. \end{array}$$

--In the above equation (9)*d*_*jz*_ represent the Euclidean distance among glowworms *j* and *z*. Finally, local decision range *rd*_*j*_ is altered using

(10) $$\begin{array}{c} rd_{j}\left(t\right)=\text{min}\left\{rs,\text{max}\left[0,rd_{j}\left(t-1\right)+\beta \left(nt-\left|N_{j}\left(t-1\right)\right|\right)\right]\right\}, \end{array}$$

where *rd*_*j*_(*t* − 1) denotes the preceding *rd*_*j*_, *r*_*s*_ indicates the radial sensor range constant, *β* represents a constant, *nt* signifies a constant variable utilized for restricting the neighborhood set size, and |*N*_*j*_(*t*)| implies the real neighborhood set size. In this presented model, the local decision range updating step can be relaxed and the values of *rd*_*j*_ are set to be the same as *r*_*s*_ constant. But, the *nt* and *β* parameters are also relaxed.

Once *X*_*i*_ is decoded for attaining centers *C*, calculate fuzzy partition *U* Matrix, and the fitness function of the ith glowworm can be determined as follows:

(11) $$\begin{array}{c} f_{i}=J_{\text{GSO}-\text{FEC}}. \end{array}$$

The minimization of *f*_*i*_ is identical to the minimization of the objective function *J*_GSO−FEC_ that resulted in optimum partition of the CT images.

### 3.3. VGG-19-Based Feature Extraction

At the time of feature extraction process, the VGG-19 model receives the segmented image as input and produces feature vectors. The VGG19 network was analogous to VGG16; however, this network would have nineteen layers rather than sixteen that consist of three FC dense layers and sixteen convolution layers. The 1st and 2nd layers have sixty-four filter of 3 × 3 kernel and pooling layers. The 2nd and 3rd convolution layers have 128 filters of 3 × 3 kernel and max pooling layers [22]. Consecutively, it has 4 convolution layers with 256 filters of 3 × 3 kernel and pooling layers. More than two sets of four convolution layers with 512 filters of 3 × 3 kernel and layers are sequentially organized. Then, this output is fed into FC layers. There are 3 FC dense layers with 1000, 4096, and 4096 neurons, respectively. The activation function was ReLu for each layer except the final dense layer in which softmax activation function was utilized.

### 3.4. Image Classification Using OMKELM Technique

At the final stage, the OMKELM model is applied for the classification process. The typical KELM is a kernel-based technique. As distinct functions provide various measures to the instance points, efficiency of various functions can be obtained significantly on the similar dataset. The ECG signals have the features of a huge volume, irregular distribution of instances produced by maximum dimension feature spaces, and imbalanced class. Utilizing a single kernel for processing ECG signals could not resolve the problem well. The kernel function was considered local or global kernel functions based on whether it is translation or rotation invariances [23]. The local kernel process was better at removing the features of instances. During the multikernel learning, an optimum kernel was assumed, that is, linear combination of the group of margins. The RBF and polynomial kernels are local and global kernel functions with optimum efficiency, respectively. The ECG signals exhibit several features, including (i) a high amount of data, (ii) an uneven distribution of instances created by maximum dimension feature spaces, and (iii) a class that is unequally distributed across the dataset. When it came to the processing of ECG signals, using a single kernel did not provide a sufficient solution to the problem. For balancing combination of the generalized capability and classifier efficiency, an MKELM was formed by linear combination of the RBF as well as polynomial kernels. The varied kernel functions are determined as

(12) $$\begin{array}{c} K_{\text{mix}}=\lambda k_{\text{rbf}}\left(u,u_{i}\right)+\left(1-\lambda \right)k_{\text{poly}}\left(u,u_{j}\right), \end{array}$$

where *λ*(0 < *λ* < 1) refers the weight coefficients of linear and its combination.

(13) $$\begin{array}{c} k_{\text{rbf}}\left(u,u_{j}\right)=\text{exp}\left(\frac{-{\left\|u-u_{i}\right\|}^{2}}{2\sigma^{2}}\right),\;\\ k_{\text{poly}}\left(u,u_{i}\right)={\left(u\cdot u_{i}+1\right)}^{d},\; \end{array}$$

where *d* refers the fixed to two, as the dimension of polynomial space is *n*^*d*^; once the instance size was equivalent to 1000 and the index was equivalent to three, the dimension is attained 1 billion. When the dimension reaches one billion, the inner product computation generates a dimension disaster [24].

At last, the resultant purpose of MKELM was determined as

(14) $$\begin{array}{c} f\left(x\right)=\left[K_{\text{mix}}\left(u,u_{1}\right),\ldots ,K_{\text{mix}}\left(u,u_{N}\right)\right]{\left(\frac{1}{C}+M\right)}^{-1}T. \end{array}$$

To optimally tune the weight parameter of the MKELM model, the COA is applied to it. The population in the COA was separated to equivalent amount of coyotes per pack. All the coyote's place was regarded as feasible solutions, and their social state (group of decision variables) signifies the main purpose. Primarily, this technique begins with arbitrarily allocated coyote places utilizing the subsequent formula.

(15) $$\begin{array}{c} X_{i}={\text{lb}}_{i}+r_{i}\times \left({\text{ub}}_{i}-\text{lb}\right), \end{array}$$

where ub_*i*_ and lb_*i*_ signify the upper and lower bounds, respectively, *r*_*i*_ refers the arbitrary number among zero and one, and *X*_*i*_ stands for the place of coyote of the *i*th dimension. In COA, the amount of coyotes per pack was restricted to 14. It can ensure the search ability of technique. An optimum coyote was determined as the optimum one modified to the environment. During the COA, the coyotes were ordered to contribute to packing maintenance and for sharing the social condition [25]. The social tendencies of pack were calculated utilizing the subsequent formula:

(16) $$\begin{array}{c} Y_{i}^{p,t}=\left\{\begin{array}{cc} C_{\left(N_{c}+1\right)/2}^{p,t},\; & N_{c}\;is\text{ odd,}\\ \frac{C_{\left(\left(N_{c}+1\right)/2\right),i}^{p,t}}{2}, & \text{otherwise,} \end{array}\right) \end{array}$$

where *N*_*c*_ refers the amount of coyotes, *Y*_*i*_^*p*,*t*^ represents the social tendencies of *p*th pack from the *t*th time, and *C* signifies the coyote-ranked social states. According to the birth and death (two important biological events of life), the birth of novel coyote was calculated dependent upon the subsequent formula:

(17) $$\begin{array}{c} B_{i}^{p,t}=\left\{\begin{array}{cc} X_{r1,i}^{p,t},\;r_{j}\geq {\mathrm{Pr}}_{s}+{\mathrm{Pr}}_{a}, & \text{or }i=i1,\\ X_{r2,i}^{p,t},\;r_{i}<{\mathrm{Pr}}_{s}, & \text{or }i=i2,\\ R_{i}, & \text{otherwise}, \end{array}\right) \end{array}$$

where *i*1 and *i*2 stands for 2 arbitrary dimensions, *r*1 and *r*2 imply the 2 coyotes arbitrarily chosen in the *p*th pack, *r*_*i*_ refers to the arbitrary number created from the range zero and one , Pr_*a*_ denotes the connection probability, and Pr_*s*_ indicates the scatter probabilities. Pr_*a*_ and Pr_*s*_ is given as

(18) $$\begin{array}{c} {\mathrm{Pr}}_{s}=\frac{1}{D},\\ {\mathrm{Pr}}_{a}=\frac{1-{\mathrm{Pr}}_{s}}{2}. \end{array}$$

During all iterations, all the *c*th coyotes from the *p*th pack upgrade their social state utilizing the succeeding formula:

(19) $$\begin{array}{c} X_{c}^{p,t+1}=\left\{\begin{array}{cc} X_{c}^{p,t}+r1\times \sigma_{1}+r2\times \sigma_{2}, & F_{c}^{p,t+1}<F_{c}^{p,t},\\ X_{c}^{p,t}, & \text{otherwise,} \end{array}\right) \end{array}$$

where *σ*_1_ and *σ*_2_ signify the alpha and pack influences, respectively. It can be determined as

(20) $$\begin{array}{c} \sigma_{1}={\text{alpha}}^{p,t}-X_{r1}^{p,t},\\ \sigma_{2}=Y^{p,t}-X_{r2}^{p,t}, \end{array}$$

where alpha^*p*,*t*^ refers the alpha coyote and *F*_*c*_^*p*,*t*^ implies the social state cost (main function). It can be computed as

(21) $$\begin{array}{c} F_{c}^{p,t+1}=f\left(X_{c}^{p,t}\right). \end{array}$$

At last, optimum coyotes are chosen dependent upon the social conditions cost as optimum solutions attained of the problems.

The COA approach develops an FF for attaining enhanced classifier efficiency. It defines a positive integer for representing the optimum efficiency of candidate solution. The error rate of the classifier was assumed to be FF (fitness function). An optimum solution has a lesser error rate and the worst solutions obtain an improved error rate:

(22) $$\begin{array}{c} \text{fitness}\left(x_{i}\right)=\text{classifier error rate}\left(x_{i}\right)\\ =\frac{\text{number of misclassified instances}}{\text{total number of instances}}*100. \end{array}$$

## 4. Performance Validation

The experimental result analysis of the AIMA-ICHDC technique uses a benchmark ICH dataset [26] from the PhysioNet repository. The dataset includes a total of 341 ICH images, including epidural class of 171 images, 24 images in intraventricular, 72 images in intraparenchymal, 56 images in subdural, and 18 images in subarachnoid. The size of images is 512*∗*512 pixels. A few sample images are illustrated in Figure 3.

A brief ICH classification result analysis of the AIMA-ICHDC technique under distinct batch size (BS) is revealed in Table 1.  Figure 4 demonstrates the result analysis of the AIMA-ICHDC technique on the ICH images under BS of 32 and varying epochs. The experimental values indicated that the AIMA-ICHDC technique has attained effective ICH detection results. For instance, with 100 epochs, the AIMA-ICHDC technique has offered sens_*y*_, spec_*f*_,  prec_*n*_, and accu_*y*_ of 93.58%, 97.94%, 95.45%, and 95.68%, respectively. Along with that, with 500 epochs, the AIMA-ICHDC technique has attained sens_*y*_, spec_*f*_,  prec_*n*_, and accu_*y*_ of 94.63%, 97.02%, 96.36%, and 96.06%, respectively.

Figure 5 depicts the result analysis of the AIMA-ICHDC approach on the ICH images under BS of 64 and varying epochs. The experimental values show that the AIMA-ICHDC algorithm has gained effectual ICH detection outcomes. For instance, with 100 epochs, the AIMA-ICHDC system has obtained sens_*y*_, spec_*f*_,  prec_*n*_, and accu_*y*_ of 93.89%, 98.67%, 96.14%, and 96.75%, respectively. Also, with 500 epochs, the AIMA-ICHDC approach has obtained sens_*y*_, spec_*f*_,  prec_*n*_, and accu_*y*_ of 94.40%, 98.38%, 96.43%, and 96.23%, respectively.

Figure 6 portrays the result analysis of the AIMA-ICHDC approach on the ICH images under BS of 128 and varying epochs. The experimental values represent that the AIMA-ICHDC methodology has effectively achieved ICH detection outcomes. For instance, with 100 epochs, the AIMA-ICHDC algorithm has obtainable sens_*y*_, spec_*f*_,  prec_*n*_, and accu_*y*_ of 95.84%, 99.11%, 96.30%, and 96.08%, respectively. At last, with 500 epochs, the AIMA-ICHDC method has reached sens_*y*_, spec_*f*_,  prec_*n*_, and accu_*y*_ of 95.49%, 97.97%, 96.55%, and 96.58%, respectively.

An average ICH result analysis of the AIMA-ICHDC technique taking place under varying BS is shown in Figure 7. On the applied BS of 32, the AIMA-ICHDC technique has depicted increased average sens_*y*_, spec_*f*_,  prec_*n*_, and accu_*y*_ of 94.09%, 97.84%, 95.82%, and 95.93%, respectively. Likewise, on the applied BS of 64, the AIMA-ICHDC system has portrayed higher average sens_*y*_, spec_*f*_,  prec_*n*_, and accu_*y*_ of 94.48%, 98.50%, 96.15%, and 96.47%, respectively. Similarly, on the applied BS of 128, the AIMA-ICHDC method has outperformed maximum average sens_*y*_, spec_*f*_,  prec_*n*_, and accu_*y*_ of 95.25%, 98.83%, 96.50%, and 96.51%, respectively.

Figure 8 shows the accuracy analysis of the AIMA-ICHDC approach on the test dataset. The outcomes outperformed that the AIMA-ICHDC method has accomplished enhanced performance with the higher training and validation accuracy. It can be revealed that the AIMA-ICHDC technique has achieved increased validation accuracy on the training accuracy.

Figure 9 demonstrates the loss analysis of the AIMA-ICHDC system on the test dataset. The results define that the AIMA-ICHDC technique has resulted in a proficient outcome with decreased training and validation loss. It can be stated that the AIMA-ICHDC methodology has presented lower validation loss on the training loss.

Table 2 provides an overall ICH detection performance analysis of the AIMA-ICHDC approach with existing techniques.

Figure 10 inspects the comparative analysis of the AIMA-ICHDC technique in terms of sens_*y*_ and spec_*y*_. The results reported that the SVM model has obtained lower values of sens_*y*_ and spec_*y*_. Besides, the WEM-DCNN and deep CNN techniques have attained slightly increased values of sens_*y*_ and spec_*y*_. Along with that, the RF model has resulted in moderate values of sens_*y*_ and spec_*y*_. Although the DL-ICH and AMG-LSTN techniques have reached reasonable values of sens_*y*_ and spec_*y*_, the proposed AIMA-ICHDC technique has shown outperforming results with the sens_*y*_ and spec_*y*_ of 95.25% and 98.83%, respectively.

Figure 11 examines the comparative analysis of the AIMA-ICHDC algorithm with respect to prec_*n*_ and acc_*y*_. The outcomes stated that the SVM method has attained lesser values of prec_*n*_ and acc_*y*_. In addition, the WEM-DCNN and deep CNN approaches have reached somewhat superior values of sens_*y*_ and spec_*y*_. Likewise, the RF technique has resulted in moderate values of prec_*n*_ and acc_*y*_. Besides, the DL-ICH and AMG-LSTN methodologies have achieved reasonable values of prec_*n*_ and acc_*y*_, and the projected AIMA-ICHDC technique has demonstrated outcomes with the prec_*n*_ and acc_*y*_ of 96.50% and 96.51%, respectively.

Finally, a computation time (CT) analysis of the AIMA-ICHDC technique with other ICH detection models is shown in Table 3 and Figure 12 [27–31]. From the figure, it can be observed that the SVM, deep CNN, and WEM-DCNN techniques have required higher CTs of 1.483 min, 1.284 min, and 1.268 min, respectively. Besides, the DL-ICH, AMG-LSN, and RF models have needed moderate CT of 0.498 min, 0.541 min, and 0.584 min, respectively. However, the AIMA-ICHDC technique has resulted in effective performance with the least CT of 0.354 min. From the results and discussion, it is ensured that the AIMA-ICHDC technique has attained maximum ICH detection and classification performance compared to existing techniques.

## 5. Conclusion

In this study, an effective AIMA-ICHDC technique has been developed with the classification and recognition of ICH using CT images. The AIMA-ICHDC technique encompasses several subprocesses such as preprocessing, GSO-FEC segmentation, feature extraction, MKELM-based classification, and COA-based parameter optimization. The design of the GSO algorithm for improving the efficiency of the FEC technique and COA to tune the parameters of the MKELM technique helps for accomplishing enhanced ICH classification performance. A lot of simulations are performed on the benchmark ICH dataset, and the results are looked at from a lot of different angles. Comparing the results, it was found that the AIMA-ICHDC strategy outperformed previous state-of-the-art ICH classification systems on a number of different factors. Using the AIMA-ICHDC approach, 0.354 minutes of CT time was saved. It is clear from the results and discussion that the AIMA-ICHDC technique has done the best job of finding and classifying ICHs than any other technique. For reporting the improvement of the AIMA-ICHDC approach, a comprehensive set of simulations are implemented utilizing the benchmark ICH dataset. Specifically, the AIMA-ICHDC technique combines glowworm swarm optimization with fuzzy entropy clustering (GSO-FEC) for the segmentation process. Additionally, the VGG-19 model was used to generate a set of feature vectors, and the optimal mixed-kernel-based extreme learning machine (OMKELM) model was used as a classifier. The coyote optimization algorithm (COA) was used to determine the ideal weight parameter for the MKELM method. Numerous simulation analyses are performed under a variety of different conditions. The AIMA-ICHDC technique's classification performance can be improved by using DL-based image segmentation algorithms in the upcoming. The extensive result analysis portrayed the supremacy of the AIMA-ICHDC technique with other techniques in terms of different measures. In future, the classification performance of the AIMA-ICHDC technique was improved with the utilization of DL-based image segmentation approaches.

## Figures and Tables

**Figure 1:** Overall working process of the AIMA-ICHDC approach.

**Figure 2:** Flowchart of GSO.

**Figure 3:** Sample images.

**Figure 4:** Result analysis of AIMA-ICHDC technique under BS of 32.

**Figure 5:** Result analysis of AIMA-ICHDC technique under BS of 64.

**Figure 6:** Result analysis of AIMA-ICHDC technique under BS of 128.

**Figure 7:** Average analysis of AIMA-ICHDC technique under distinct BS.

**Figure 8:** Accuracy graph analysis of AIMA-ICHDC technique.

**Figure 9:** Loss graph analysis of AIMA-ICHDC technique.

**Figure 10:** Sens_*y*_ and Spec_*y*_ analysis of AIMA-ICHDC technique with existing approaches.

**Figure 11:** Prec_*n*_ and Acc_*y*_ analysis of AIMA-ICHDC technique with existing approaches.

**Figure 12:** CT analysis of AIMA-ICHDC algorithm with other ICH detection methods.

**Table 1:** Result analysis of AIMA-ICHDC technique under varying batch size.

No. of epochs	Sensitivity	Specificity	Precision	Accuracy
Batch size = 32				
100	93.58	97.94	95.45	95.68
200	93.38	98.09	95.43	95.93
300	94.32	98.02	95.44	95.69
400	94.53	98.11	96.43	96.27
500	94.63	97.02	96.36	96.06
Average	**94.09**	**97.84**	**95.82**	**95.93**
Batch size = 64				
100	93.89	98.67	96.14	96.75
200	93.89	98.55	95.95	96.31
300	94.34	98.20	96.08	96.41
400	95.90	98.70	96.15	96.65
500	94.40	98.38	96.43	96.23
Average	**94.48**	**98.50**	**96.15**	**96.47**
Batch size = 128				
100	95.84	99.11	96.30	96.08
200	95.70	99.19	96.93	96.31
300	93.90	99.17	96.73	96.86
400	95.30	98.71	96.00	96.72
500	95.49	97.97	96.55	96.58
Average	**95.25**	**98.83**	**96.50**	**96.51**

**Table 2:** Comparative analysis of AIMA-ICHDC technique with existing approaches.

Methods	Sensitivity	Specificity	Precision	Accuracy
AIMA-ICHDC	95.25	98.83	96.50	96.51
DL-ICH	94.22	97.60	95.57	95.58
AMG-LSN	92.07	93.57	93.77	92.95
Random forest	90.68	89.63	89.30	89.99
WEM-DCNN	83.61	97.83	90.51	88.38
Deep CNN	87.88	88.51	88.69	88.25
SVM model	76.44	79.63	78.38	77.58

**Table 3:** CT analysis of AIMA-ICHDC technique with other ICH detection models.

Methods	Computation time (min)
AIMA-ICHDC	0.354
DL-ICH	0.498
AMG-LSN	0.541
Random forest	0.584
WEM-DCNN	1.268
Deep CNN	1.284
SVM model	1.483

## Data Availability

No data were used to support this study.
